The article "Dexmedetomidine Alleviates Lung Oxidative Stress Injury Induced by Ischemia-Reperfusion in Diabetic Rats via the Nrf2-Sulfiredoxin1 Pathway" was published in 2022. Journal: Biomed Res Int.

# Dexmedetomidine Alleviates Lung Oxidative Stress Injury Induced by Ischemia-Reperfusion in Diabetic Rats via the Nrf2-Sulfiredoxin1 Pathway

**DOI:** 10.1155/2022/5584733

**Published:** 2022-02-24

**Authors:** Xuan Wang, Bing Zhang, Guangqi Li, Han Zhao, Xiaojun Tian, Junmin Yu, Yanwei Yin, Chao Meng

**Affiliations:** ^1^Department of Anesthesiology, The Affiliated Hospital of Qingdao University, Qingdao, China 266000; ^2^Department of Pathology, The Affiliated Hospital of Qingdao University, Qingdao, China 266000; ^3^Department of Radiology, The Affiliated Hospital of Qingdao University, Qingdao, China 266000; ^4^Department of Pain Management, The Affiliated Hospital of Qingdao University, Qingdao, China 266000

## Abstract

Oxidative stress injury (OSI) is an important pathological process in lung ischemia-reperfusion injury (LIRI), and diabetes mellitus (DM) can exacerbate this injury. Dexmedetomidine protects against LIRI by reducing OSI. However, the effect of dexmedetomidine on LIRI under diabetic conditions remains unclear. Therefore, this study is aimed at exploring the effects and mechanisms of dexmedetomidine on OSI induced by LIRI in diabetic rats. Rats were randomly divided into control+sham (CS), DM+sham (DS), control+ischemia-reperfusion (CIR), DM+ischemia-reperfusion (DIR), and DM+ischemia-reperfusion+dexmedetomidine (DIRD) groups (*n* = 6). In the CS and DS groups, the nondiabetic and diabetic rats underwent thoracotomy only without LIRI. In the CIR, DIR, and DIRD groups, LIRI was induced through left hilum occlusion for 60 min, followed by reperfusion for 120 min in nondiabetic and diabetic rats, and rats in the DIRD group were administered dexmedetomidine (3, 5, and 10 *μ*g/kg). Compared with those in the CS group, the OSI, lung compliance, apoptosis, and oxygenation indices deteriorated in the DS group (*P* < 0.05), and these indices were further aggravated in the CIR and DIR groups (*P* < 0.05), being the worst in the DIR group (*P* < 0.05). Compared to those of the DIR group, the OSI, lung compliance (15.8 ± 2.4 vs. 11.6 ± 1.7 ml/kg), apoptosis (22.5 ± 2.6 vs. 51.8 ± 5.7), oxygenation (381 ± 58 vs. 308 ± 78 mmHg), and caspase-3 and caspase-9 protein expression indices were attenuated, and Nrf2 and sulfiredoxin1 protein expression was increased in the DIRD group (*P* < 0.05). And the lung injury, oxygenation, OSI, and Nrf2 and sulfiredoxin1 protein expression changed in a concentration-dependent manner. In conclusion, dexmedetomidine alleviated lung OSI and improved lung function in a diabetic rat LIRI model through the Nrf2-sulfiredoxin1 pathway.

## 1. Introduction

Many people have diabetes mellitus (DM) worldwide. With an increased occurrence in both aging individuals and young adults (<40 years old), DM is an independent risk factor for morbidity and mortality after lung ischemia-reperfusion (I/R) injury, especially in those with type 2 DM [1]. DM is associated with many severe complications, and the lung is one of the target organs [2]. In the context of diabetes, increased attention should be paid to preventing lung injury during lung surgery.

The article "Dexmedetomidine Alleviates Lung Oxidative Stress Injury Induced by Ischemia-Reperfusion in Diabetic Rats via the Nrf2-Sulfiredoxin1 Pathway" was published in 2022. Journal: Biomed Res Int.

Lung I/R injury can occur in many clinical contexts, such as lung transplantation, shock, cardiopulmonary bypass, and single-lung ventilation, which can contribute to severe organ failure and increase mortality in patients [3, 4]. Oxidative stress injury can lead to the intracellular generation of reactive oxygen species (ROS), which are important factors that contribute to lung I/R injury [5]. Additionally, previous studies have shown that sustained hyperglycemia produces excessive ROS, which contribute to diabetic lung injury in rats and humans [6–9]. Thus, the inhibition of oxidative stress injury is essential for alleviating diabetic lung I/R injury.

Dexmedetomidine (DEX), a highly selective *α*_2_-adrenergic agonist with sedative, anxiolytic, analgesic, and sympatholytic inhibitory characteristics, has been widely applied in the clinic [10]. Although DEX has been shown to have protective effects on lung I/R injury by decreasing oxidative stress injury, the specific mechanism by which DEX affects oxidative stress injury remains unclear [11, 12]. A previous study showed that nuclear factor erythroid 2-related factor (Nrf2) and its downstream protein sulfiredoxin1 participated in oxidative stress injury [13]. DEX pretreatment could activate the Nrf2 pathway in many organs in I/R models, such as the liver, brain, and intestines [14–16]. However, whether the effects of DEX on diabetic lung I/R injury are related to Nrf2-sulfiredoxin1-induced antioxidative effects is still unknown. Through this study, we provided an innovative pathway, Nrf2-sulfiredoxin1 pathway, and tried to explain its effects on oxidative stress injury induced by lung I/R. Therefore, this study is aimed at examining the effects of DEX on lung injury induced by I/R in diabetic rats and exploring the potential role of the Nrf2-sulfiredoxin1 pathway. We present this article in accordance with the ARRIVE checklist.

## 2. Materials and Methods

### 2.1. Animals

Adult, pathogen-free male Sprague Dawley rats weighing 200-220 g were purchased from the Experiment Center of the Affiliated Hospital of Qingdao University. The animals were housed in a temperature-controlled room with ad libitum access to food and water and a 12-12 h light-dark cycle before the experiment. The animal health and behavior were monitored every day. The Animal Care and Welfare Committee approved all experiments and procedures in this study (No. AHQU-MAL20180913).

The article "Dexmedetomidine Alleviates Lung Oxidative Stress Injury Induced by Ischemia-Reperfusion in Diabetic Rats via the Nrf2-Sulfiredoxin1 Pathway" was published in 2022. Journal: Biomed Res Int.

### 2.2. DM Model

The DM rat model was established by the administration of a high-fat diet (15% lard, 5% sesame oil, 20% sucrose, 2.5% cholesterol, and 57.5% normal chow) for 4 weeks followed by a low-dose intraperitoneal injection of streptozotocin (35 mg/kg, dissolved to a concentration of 0.1 M, pH 4.5, Sigma-Aldrich; Merck KGaA, Darmstadt, Germany). A fasting blood glucose level ≥ 11.1 mmol/l at 72 h after streptozotocin injection was considered indicative of DM [17]. The rats fed a standard diet were used as nondiabetic controls.

### 2.3. Lung I/R Injury Model

The rats were anesthetized by an intraperitoneal injection of sodium pentobarbital (60 mg/kg). After anesthesia, the rats were intubated with a tracheal tube under a laryngoscope. The tracheal tube was connected to a small animal ventilator for mechanical ventilation with a tidal volume of 8 ml/kg. The respiratory rate was adjusted to maintain an arterial carbon dioxide tension (PaCO_2_) of 35-45 mmHg. The femoral artery and vein were cannulated for blood pressure monitoring and drug administration, respectively. After a left lateral thoracotomy, the left lung hilum was clamped 5 min after the administration of heparin (50 IU/animal) with a noninvasive microvascular clip at the end of expiration. The tidal volume was reduced to 6 ml/kg during clamping. After a 60 min ischemic period, the microvascular clip was removed for 120 min of reperfusion. Then, the tidal volume was adjusted to 8 ml/kg. During the experiment, the body temperature was maintained between 37.5°C and 38.5°C with a heating blanket. At the end of the experiment, the rats were euthanized by exsanguination under anesthesia.

### 2.4. Groups

The rats were randomly divided into 5 groups (*n* = 6): control+sham (CS) group, DM+sham (DS) group, control+I/R (CIR) group, DM+I/R (DIR) group, and DM+I/R+DEX (DIRD) group. In order to further explore the effects of DEX, 3 *μ*g/kg, 5 *μ*g/kg, and 10 *μ*g/kg were used. In the CS and DS groups, the nondiabetic and diabetic rats underwent thoracotomy and were ventilated with 40% O_2_ without ischemia and reperfusion. In the CIR and DIR groups, lung I/R injury was established in the nondiabetic and diabetic rats, which were then ventilated with 40% O_2_. In the DIRD group, lung I/R injury was established in diabetic rats, and DEX (No. 191005BP, Jiangsu Hengrui Pharmaceutical Co., Ltd., Lianyungang, China) was administered through the femoral vein for 10 min before reperfusion. The rats in the other groups were administered the same volume of normal saline (Figure 1).

The article "Dexmedetomidine Alleviates Lung Oxidative Stress Injury Induced by Ischemia-Reperfusion in Diabetic Rats via the Nrf2-Sulfiredoxin1 Pathway" was published in 2022. Journal: Biomed Res Int.

### 2.5. Blood Gas Analysis

Arterial blood gas analysis was performed by a blood gas analyzer (Rapid Lab 248, Bayer, Medfield, MA, USA) at baseline (3 min after ventilation), 60 min after ischemia, and 60 and 120 min after reperfusion, and the data were recorded as T0-T3. At the end of the experiment, blood from the left pulmonary vein was also collected for blood gas analysis.

### 2.6. Measurement of Lung Static Compliance

After the euthanasia of the rats, the median sternotomies were immediately performed. The lungs were isolated with a tracheal tube, and the right lung hilum was ligated. Then, the tracheal tube was connected to an apparatus to measure the left lung static pressure-volume (P-V) curve to assess static lung compliance. Airway pressure was increased to 30 cm H_2_O before being decreased to 0 cm H_2_O in stepwise intervals of 5 cm. After 1 min of stabilization, the lung volume was recorded through gas compression [18]. This parameter was examined by a researcher who was blinded to the study conditions.

### 2.7. Measurement of Oxidative Stress Injury Parameters

After the euthanasia of the rats, one part of the lower lobe of the left lung was homogenized with cold normal saline to determine the 8-hydroxydeoxyguanosine (8-OHdG) level (AmyJet Scientific Inc., Wuhan, China), inducible nitric oxide synthase (iNOS) level (CUSABIO BIOTECH Co. Ltd., Wuhan, China), glutathione peroxidase (GSH-PX) activity (Beyotime Biotechnology, Shanghai, China), malondialdehyde (MDA) level (Beyotime Biotechnology, Shanghai, China), superoxide dismutase (SOD) activity (Beyotime Biotechnology, Shanghai, China), and total antioxidant capacity (T-AOC) (Beyotime Biotechnology, Shanghai, China) using commercial kits.

### 2.8. Histopathological Examination and Scoring

After the euthanasia of the rats, the middle lobe of the left lung was fixed in paraformaldehyde, embedded in paraffin, and cut into 6 *μ*m thick sections for hematoxylin-eosin (H&E) staining. The lung injury score (LIS) [19] was evaluated by histopathology based on the following criteria: (1) neutrophil infiltration, (2) airway epithelial cell damage, (3) interstitial edema, (4) hyaline membrane formation, and (5) hemorrhage. Each criterion had five scores as follows: normal = 0, minimal change = 1, mild change = 2, moderate change = 3, and severe change = 4. All sections were evaluated via light microscopy by a pathologist who was blinded to this study.

### 2.9. Apoptosis Measurement by Immunohistochemistry

The tissues, middle lobe of the left lung, embedded in paraffin were used for terminal deoxynucleotidyl transferase dUTP nick end-labeling (TUNEL) staining to assess alveolar epithelial cell apoptosis (Zhongshan Golden Bridge Biotechnology, Beijing, China). The number of positive cells per 100 cells in five random fields from the same TUNEL-stained section was counted and recorded as the apoptotic index (AI) [20]. The protein expression levels of caspase-3 and caspase-9 in lung tissues were measured using immunohistochemical staining (Zhongshan Golden Bridge Biotechnology, Beijing, China). The number of positive cells per section was counted in five random fields in each specimen to calculate the immunohistochemical score (IHS), which was determined by multiplying the quantity score (an estimation of the percentage of immunoreactive cells: no staining was scored as 0; 1%-10% of cells was scored as 1; 11%-50% was scored as 2; 51%-80% was scored as 3; and 81%-100% was scored as 4) by the staining intensity score (an estimation of the staining intensity: 0 = negative, 1 = weak, 2 = moderate, and 3 = strong). All sections were examined by a pathologist using a single-blind method [21].

The article "Dexmedetomidine Alleviates Lung Oxidative Stress Injury Induced by Ischemia-Reperfusion in Diabetic Rats via the Nrf2-Sulfiredoxin1 Pathway" was published in 2022. Journal: Biomed Res Int.

### 2.10. Western Blot Analysis

Another part of lower lobe of the left lung was homogenized in lysis buffer for protein collection. After the protein concentration was measured by a BCA kit (Beyotime Biotechnology, Shanghai, China), 50 *μ*g protein samples were separated by sodium dodecyl sulfate polyacrylamide gel electrophoresis and transferred onto a PVDF membrane. The membrane was incubated with primary antibodies against Nrf2 (1 : 3000, Santa Cruz Biotechnology, Germany) and sulfiredoxin1 (1 : 2000, Santa Cruz Biotechnology, Germany) after blocking in 5% nonfat dry milk. Then, the membrane was incubated overnight at 4°C and washed and incubated with secondary antibody (1 : 5000, Zhongshan Golden Bridge Biotechnology, Beijing, China) at room temperature for 1 h. Next, the proteins were visualized with enhanced chemiluminescence reagent (GE Healthcare Bio Sciences, Pittsburgh, PA, USA), quantified using ImageJ version 1.61 software (National Institutes of Health, Bethesda, MD, USA), and normalized to *β-*actin.

### 2.11. Statistical Analysis

Statistical testing was performed with SPSS 20.0 software. The data are expressed as the means ± standard deviation (SD). Differences among groups were assessed by one-way analysis of variance (ANOVA) followed by the Bonferroni test. Time-dependent differences were assessed through repeated analysis of variance followed by Dunnett's test. The nonparametric Kruskal Wallis test was used for the analysis of LIS and IHS data followed by the Nemenyi test. A value of *P* < 0.05 was considered indicative of statistical significance.

## 3. Results

### 3.1. Experiment-Related Data

All rats were operated on successfully in this study. After the microvascular clip was removed, the chest was closed. Thus, the total time the chest was open was 62.3 ± 1.5 min in the CS group, 62.5 ± 1.0 min in the DS group, 63.5 ± 1.0 min in the CIR group, 63.7 ± 1.0 min in the DIR group, and 63.7 ± 1.6 min in the 3 *μ*g DIRD group, 65.2 ± 1.5 min in the 5 *μ*g DIRD group, and 63.0 ± 2.5 min in the 10 *μ*g DIRD group. There were no significant differences among the groups. Additionally, the baseline data including weight (214 ± 4 g in the CS group, 214 ± 5 g in the DS group, 210 ± 8 g in the CIR group, 209 ± 5 g in the DIR group, and 211 ± 6 g in the 3 *μ*g DIRD group, 211 ± 5 g in the 5 *μ*g DIRD group, and 209 ± 7 g in the 10 *μ*g DIRD group) and blood gas analysis in all groups showed no significant differences (Table 1).

The article "Dexmedetomidine Alleviates Lung Oxidative Stress Injury Induced by Ischemia-Reperfusion in Diabetic Rats via the Nrf2-Sulfiredoxin1 Pathway" was published in 2022. Journal: Biomed Res Int.

### 3.2. DEX Improved Blood Gas Parameters

The oxygenation index (the partial pressure of arterial oxygen (PaO_2_)/fraction of inspired oxygen (FiO_2_)) at T0-T3 in the CS and DS groups was stable. At the T0 time point, the oxygenation indices in all groups were not significantly different. At the T1 time point, the oxygenation index in the CIR, DIR, and DIRD groups was significantly decreased compared with that in the CS and DS groups (*P* < 0.05). At the T2 time point, compared with that in the CS group, the oxygenation index decreased significantly in the DS, CIR, DIR, and DIRD groups (*P* < 0.05). Compared with that in the DS group, the oxygenation index in the CIR, DIR, and DIRD groups was further decreased, and the oxygenation index in the DIR group was lower than that in the CIR group (*P* < 0.05). Compared with that in the DIR group, the oxygenation index in the DIRD group was increased significantly (*P* < 0.05). The oxygenation index in all groups at the T3 time point exhibited a similar trend as that at T2, as did the base excess and pH values (Table 1). Additionally, there was also a similar trend in the analysis of blood from the left pulmonary vein as the related indices shown above, which provided concentration-dependent effects (Table 2 and Figure 2).

### 3.3. DEX Improved Lung Static Compliance

Compared with those in the CS group, the P-V curve values in the DS, CIR, DIR, and DIRD groups were lower, and the values in the CIR, DIR, and DIRD groups were markedly lower than those in the DS group (*P* < 0.05). Compared with that in the CIR group, the P-V curve value in the DIR group was further decreased (*P* < 0.05). However, the value in the DIRD group was higher than that in the DIR group (*P* < 0.05). At a pressure of 30 cm H_2_O, the values in the CS, DS, CIR, DIR, and DIRD groups were 18.3 ± 1.0 ml/kg, 17.1 ± 0.7 ml/kg, 13.3 ± 0.9 ml/kg, 11.5 ± 1.3 ml/kg, and 15.5 ± 0.8 ml/kg, respectively (Figure 3).

The article "Dexmedetomidine Alleviates Lung Oxidative Stress Injury Induced by Ischemia-Reperfusion in Diabetic Rats via the Nrf2-Sulfiredoxin1 Pathway" was published in 2022. Journal: Biomed Res Int.

### 3.4. DEX Maintained Lung Tissue Structure

The histological changes showed minimal lung injury in the CS group, mild lung injury in the DS group, and severe lung injury in the CIR and DIR groups. In contrast, the histological changes showed moderate damage in the DIRD group. The LISs paralleled the histological changes. Therefore, the neutrophil infiltration LIS in the DS group (0.5 (0 to 2)) was higher than that in the CS group (0 (0 to 1)), and the neutrophil infiltration LIS in the CIR group (3 (1 to 3)) was higher than that in the CS and DS groups (*P* < 0.05). The neutrophil infiltration LIS in the DIR group (4 (3 to 4)) was higher than that in the CIR group, and the neutrophil infiltration LIS in the DIRD group (1.5 (1 to 2)) was lower than that in the DIR group (*P* < 0.05). The LISs of the other criteria also exhibited similar trends (Figure 4). Additionally, the lung injury score improved in a concentration-dependent manner (Figure 5).

### 3.5. DEX Decreased Lung Oxidative Stress Injury

Compared with that in the CS and DS groups, the MDA level was significantly increased in the CIR, DIR, and DIRD groups, and the MDA level in the DS group was higher than that in the CS group (*P* < 0.05). Compared with that in the CIR and DIR groups, the MDA level in the DIRD group was significantly decreased, and the MDA level in the DIR group was higher than that in the CIR group (*P* < 0.05). The levels of 8-OHdG and iNOS showed the same trend as those of MDA (*P* < 0.05). Additionally, the activities of GSH-PX, SOD, and T-AOC showed the opposite trend to those of MDA (*P* < 0.05) (Table 3). Additionally, the oxidative stress injury changed in a concentration-dependent manner (Figure 6).

### 3.6. DEX Decreased Apoptosis in Lung Tissue

Compared with that in the CS and DS groups, the number of TUNEL-positive cells in the CIR, DIR, and DIRD groups increased significantly, and the number of TUNEL-positive cells in the DS group was higher than that in the CS group (*P* < 0.05). Compared with that in the CIR and DIR groups, the number of TUNEL-positive cells in the DIRD group was significantly decreased, and the number in the DIR group was higher than that in the CIR group (*P* < 0.05). Therefore, compared with that in the CS (6.3 ± 2.5) and DS groups (14.8 ± 2.6), the AI in the CIR group (38.8 ± 6.9), the DIR group (51.8 ± 5.7), and the DIRD group (22.5 ± 2.6) was significantly increased (*P* < 0.05). Compared with that in the CIR and DIR groups, the AI in the DIRD group was significantly decreased, and the AI in the DIR group was higher than that in the CIR group (*P* < 0.05) (Figure 7). Additionally, a similar trend was observed in the IHS of caspase-3 and caspase-9 (Figures 8 and 9).

The article "Dexmedetomidine Alleviates Lung Oxidative Stress Injury Induced by Ischemia-Reperfusion in Diabetic Rats via the Nrf2-Sulfiredoxin1 Pathway" was published in 2022. Journal: Biomed Res Int.

### 3.7. DEX Activated the Nrf2-Sulfiredoxin1 Pathway

Compared with those in the CS and DS groups, the Nrf2 and sulfiredoxin1 protein expression levels in the CIR and DIR groups were increased significantly (*P* < 0.05), and the Nrf2 and sulfiredoxin1 protein expression levels in the DIRD group were significantly increased compared with those in the DIR and CIR groups (*P* < 0.05) (Figure 10). Additionally, the Nrf2 and sulfiredoxin1 protein expression levels increased in a concentration-dependent manner (Figure 11).

## 4. Discussion

In this study, DM exacerbated lung I/R injury in rats, as demonstrated by decreases in oxygenation, lung compliance, GSH-PX, SOD, and T-AOC; severe tissue structure damage; and increases in 8-OHdG, iNOS, MDA, and apoptosis. The administration of DEX before reperfusion alleviated lung I/R injury, maintained oxygenation and lung compliance, and decreased apoptosis by increasing antioxidant capacity and reducing oxidative stress injury. Additionally, DEX activated the Nrf2-sulfiredoxin1 pathway, which was associated with the protective effects of DEX on diabetic lung I/R injury.

Oxidative stress injury is the initial mechanism of I/R injury [22]. MDA is one of the most important products of membrane lipid peroxidation, 8-OHdG is the most commonly used biomarker of DNA oxidative damage, and iNOS induces a large amount of NO and causes oxidative stress injury when stimulated. SOD is an antioxidative metal enzyme, T-AOC is an indicator of the total antioxidative level, and GSH-PX is an important peroxidase that protects the cell membranes from peroxide damage. This study evaluated oxidative stress through these indices. Oxidative stress injury could lead to the intracellular generation of ROS, which directly leads to tissue injury and apoptosis [23]. The resultant oxidant stress has been implicated in the subsequent development of the inflammatory response, which increases apoptosis and decreases lung compliance and oxygenation [24]. In this study, severe oxidative stress injury was found, and worsened tissue structure, compliance, oxygenation function, and apoptosis were also observed after reperfusion, which was consistent with the findings of previous studies [25–27].

DM, characterized by persistent blood hyperglycemia, was related to approximately 1.5 million deaths in 2012 [2]; moreover, DM is an independent risk factor for morbidity and mortality after lung I/R injury [1]. We hypothesized that DM was associated with oxidative stress injury. First, hyperglycemia can induce the overproduction of superoxide in many kinds of tissue injuries [28]. Second, sustained hyperglycemia produces excessive ROS, resulting in damage to DNA, lipids, and proteins [6, 29]. In this study, we also found that DM worsened lung I/R injury and induced excessive oxidative stress injury, which was also demonstrated by other studies [4, 30]. Therefore, reducing oxidative stress injury is important for the treatment of diabetic lung I/R injury.

The article "Dexmedetomidine Alleviates Lung Oxidative Stress Injury Induced by Ischemia-Reperfusion in Diabetic Rats via the Nrf2-Sulfiredoxin1 Pathway" was published in 2022. Journal: Biomed Res Int.

DEX, a second-generation, highly selective *α*_2_-adrenergic receptor agonist, is used as a preoperative sedative and general anesthesia adjuvant in the clinic. In 2017, Fu et al. [31] showed that DEX decreased lipopolysaccharide-induced acute lung injury by regulating the levels of ROS and lipid peroxides. In 2018, Zhou et al. [32] reported that DEX could attenuate MDA levels and improve SOD levels to decrease oxidative stress injury in a rat ex vivo lung I/R model. In 2019, Liang et al. [11] also demonstrated that DEX decreased lung I/R injury by decreasing oxidative stress injury. Considering the antioxidative effects of DEX, we hypothesized that DEX could also exert a beneficial effect in diabetes models. Thus, this study applied DEX in a model of DM. The results showed that DEX reduced oxidative stress injury, decreased apoptosis, maintained cell structure stability, and improved lung function. These effects were concentration dependent. This finding further confirmed our initial hypothesis.

Although the protective effects of DEX on lung I/R injury have been recognized, the mechanisms remain unclear. In 2017, Wu et al. [33] found that sulfiredoxin1 could prevent cerebral I/R-induced oxidative stress injury. In 2018, Zhang et al. [13] demonstrated that when Nrf2 expression decreased, its downstream protein, sulfiredoxin1, was decreased in an oxygen-glucose deprivation/reoxygenation model in primary neurons, and oxidative stress injury was exacerbated. Thus, we hypothesized that the activation of the Nrf2-sulfiredoxin1 pathway may decrease oxidative stress injury induced by lung I/R and attenuate lung I/R injury. In this study, DEX activated the protein expression of Nrf2 and sulfiredoxin1 and decreased the oxidative stress injury induced by I/R. And with the increased concentration of DEX, the more protein expressions of Nrf2 and sulfiredoxin1 were activated and the less oxidative stress injury was displayed. Through this study, we demonstrated the importance of the Nrf2-sulfiredoxin1 pathway in the protective effects of DEX on diabetic lung I/R injury.

We know that activation of Nrf2 protects against oxidative stress injury induced by ischemia-reperfusion injury. Previous studies [14, 16, 34] found that DEX restores the decline of Nrf2 activity induced by I/R injury or inflammation to the level of the control group. In their studies, the Nrf2 expression decreased in the “injury” group and DEX restores the decline of Nrf2 activity to the level of the control group, which was not exactly the same as our current research. The reasons existed. First, in the normal tissues without injury, the Nrf2 was expressed relatively low in a certain degree, while the Nrf2 expression increased in the injured tissues. This may mean a kind of self-regulation after tissue injury, and self-regulation may have a certain limit. After DEX was used, Nrf2 was further activated. So the activation of Nrf2 was much more enhanced in the DEX group than in the control group. Second, it cannot be ruled out that it was related to the conditions of the rats, the establishment of the model, the degree of tissue damage, etc. The researches of Chen et al. [15] and ours [35] provided similar results with this study. Of course, these all need to be further verified and confirmed in our future research.

The article "Dexmedetomidine Alleviates Lung Oxidative Stress Injury Induced by Ischemia-Reperfusion in Diabetic Rats via the Nrf2-Sulfiredoxin1 Pathway" was published in 2022. Journal: Biomed Res Int.

There were some limitations to the present study. First, the DEX used in nondiabetic rats was not observed. In this study, we mainly observed the effect of DEX under diabetic condition, and there have been many articles that have confirmed the protective effects of DEX on I/R injury in the lungs of normal rats [11, 12, 36]. In the future, we will explore the effects of DEX at different concentrations in the normal and diabetic I/R injury groups to clarify whether the effect of DEX is simply to reduce I/R injury or whether it is specifically effective for I/R injury enhanced by diabetes. Second, the time-dependent effects of DEX on oxidative stress injury and protein expression were not measured, so the extent of the effect of DEX is unknown. Third, this DM model was established via a straightforward procedure to simulate the clinical symptoms of diabetic patients, but these symptoms could not be fully simulated. Then, HO-1 is a widely studied downstream target of Nrf2, and the relationship between sulfredoxin1 and HO-1 will be explored in the further, which will be more conducive to the research of the Nrf2 pathway. Finally, the Nrf2-knockout model will further demonstrate the mechanism by which DEX affects lung I/R injury in diabetic rats.

## 5. Conclusions

Rat lung I/R can result in oxidative stress injury, apoptosis, and worsened lung function, and DM can exacerbate these injuries. DEX treatment can alleviate diabetic lung I/R injury by decreasing oxidative stress injury, probably via the Nrf2-sulfiredoxin1 pathway.

## Figures and Tables

**Figure 1:** Study design. (a) Rats were treated in normal and diabetic condition. (b) Under diabetic condition, different doses of DEX were used. In the DIRD group, the 3 *μ*g/kg of DEX was given. DEX: dexmedetomidine.

The article "Dexmedetomidine Alleviates Lung Oxidative Stress Injury Induced by Ischemia-Reperfusion in Diabetic Rats via the Nrf2-Sulfiredoxin1 Pathway" was published in 2022. Journal: Biomed Res Int.

**Figure 2:** The indices of blood gas analysis from pulmonary vein in different concentrations of DEX groups (mean ± SD, *n* = 6). PvO_2_/FiO_2_: pulmonary venous oxygen tension (PvO_2_)/fraction of inspired oxygen (FiO_2_); BE: base excess; DIR: diabetes mellitus+ischemia-reperfusion; 3 *μ*g DIRD: diabetes mellitus+ischemia-reperfusion+3 *μ*g/kg dexmedetomidine; 5 *μ*g DIRD: diabetes mellitus+ischemia-reperfusion+5 *μ*g/kg dexmedetomidine; 10 *μ*g DIRD: diabetes mellitus+ischemia-reperfusion+10 *μ*g/kg dexmedetomidine. ^†^*P* < 0.05 vs. the DIR group; ^‡^*P* < 0.05 vs. the 3 *μ*g DIRD group; ^┼^*P* < 0.05 vs. the 5 *μ*g DIRD group.

**Figure 3:** Lung static compliance (*n* = 6). After 120 min of reperfusion, the lungs were used to determine static compliance by pressure-volume (P-V) curves. The data are presented as the mean values, and the bars are omitted for clarity. CS: control+sham; DS: diabetes mellitus+sham; CIR: control+ischemia-reperfusion; DIR: diabetes mellitus+ischemia-reperfusion; DIRD: diabetes mellitus+ischemia-reperfusion+dexmedetomidine. In the DIRD group, the 3 *μ*g/kg of DEX was used. ^∗^*P* < 0.05 vs. the CS group; ^#^*P* < 0.05 vs. the DS group; ^△^*P* < 0.05 vs. the CIR group; ^§^*P* < 0.05 vs. the DIR group.

**Figure 4:** Pathological changes in lung tissue (original magnification, ×20). Paraformaldehyde-fixed sections of lung grafts were stained with hematoxylin and eosin. Diabetes mellitus induced lung injury and exacerbated lung ischemia-reperfusion injury. Dexmedetomidine could alleviate this lung injury. (a) CS group; (b) DS group; (c) CIR group; (d) DIR group; (e) DIRD group; (f) lung injury score (*n* = 4). CS: control+sham; DS: diabetes mellitus+sham; CIR: control+ischemia-reperfusion; DIR: diabetes mellitus+ischemia-reperfusion; DIRD: diabetes mellitus+ischemia-reperfusion+dexmedetomidine. In the DIRD group, the 3 *μ*g/kg of DEX was used. ^∗^*P* < 0.05 vs. the CS group; ^#^*P* < 0.05 vs. the DS group; ^△^*P* < 0.05 vs. the CIR group; ^§^*P* < 0.05 vs. the DIR group.

**Figure 5:** Lung pathological changes in different concentrations of DEX groups (original magnification, ×20). (a) DIR group; (b) 3 *μ*g DIRD group; (c) 5 *μ*g DIRD group; (d) 10 *μ*g DIRD group; (e) lung injury score (*n* = 4). DIR: diabetes mellitus+ischemia-reperfusion; 3 *μ*g DIRD: diabetes mellitus+ischemia-reperfusion+3 *μ*g/kg dexmedetomidine; 5 *μ*g DIRD: diabetes mellitus+ischemia-reperfusion+5 *μ*g/kg dexmedetomidine; 10 *μ*g DIRD: diabetes mellitus+ischemia-reperfusion+10 *μ*g/kg dexmedetomidine. ^†^*P* < 0.05 vs. the DIR group; ^‡^*P* < 0.05 vs. the 3 *μ*g DIRD group; ^┼^*P* < 0.05 vs. the 5 *μ*g DIRD group.

The article "Dexmedetomidine Alleviates Lung Oxidative Stress Injury Induced by Ischemia-Reperfusion in Diabetic Rats via the Nrf2-Sulfiredoxin1 Pathway" was published in 2022. Journal: Biomed Res Int.

**Figure 6:** Oxidative stress injury in different concentrations of DEX groups (mean ± SD, *n* = 6). DIR: diabetes mellitus+ischemia-reperfusion; 3 *μ*g DIRD: diabetes mellitus+ischemia-reperfusion+3 *μ*g/kg dexmedetomidine; 5 *μ*g DIRD: diabetes mellitus+ischemia-reperfusion+5 *μ*g/kg dexmedetomidine; 10 *μ*g DIRD: diabetes mellitus+ischemia-reperfusion+10 *μ*g/kg dexmedetomidine. ^†^*P* < 0.05 vs. the DIR group; ^‡^*P* < 0.05 vs. the 3 *μ*g DIRD group; ^┼^*P* < 0.05 vs. the 5 *μ*g DIRD group.

**Figure 7:** Alveolar epithelial cell apoptosis was demonstrated by TUNEL staining (original magnification, ×40). TUNEL-positive cells were observed under a light microscope and identified by brown-stained nuclei (shown with arrows). TUNEL: terminal deoxynucleotidyl transferase dUTP nick end-labeling; (a) CS group; (b) DS group; (c) CIR group; (d) DIR group; (e) DIRD group; (f) apoptosis index (*n* = 4). In the DIRD group, the 3 *μ*g/kg of DEX was used. ^∗^*P* < 0.05 vs. the CS group; ^#^*P* < 0.05 vs. the DS group; ^△^*P* < 0.05 vs. the CIR group; ^§^*P* < 0.05 vs. the DIR group.

**Figure 8:** Protein expression of caspase-3 in lung tissues by immunohistochemistry (original magnification, ×40). Caspase-3-positive cells were observed under a light microscope and identified by brown-stained nuclei. (a) CS group; (b) DS group; (c) CIR group; (d) DIR group; (e) DIRD group; (f) immunohistochemical scores (IHS) (*n* = 4). In the DIRD group, the 3 *μ*g/kg of DEX was used. ^∗^*P* < 0.05 vs. the CS group; ^#^*P* < 0.05 vs. the DS group; ^△^*P* < 0.05 vs. the CIR group; ^§^*P* < 0.05 vs. the DIR group.

**Figure 9:** Protein expression of caspase-9 in lung tissues by immunohistochemistry (original magnification, ×40). Caspase-9-positive cells were observed under a light microscope and identified by brown-stained nuclei. (a) CS group; (b) DS group; (c) CIR group; (d) DIR group; (e) DIRD group; (f) immunohistochemical scores (IHS) (*n* = 4). In the DIRD group, the 3 *μ*g/kg of DEX was used. ^∗^*P* < 0.05 vs. the CS group; ^#^*P* < 0.05 vs. the DS group; ^△^*P* < 0.05 vs. the CIR group; ^§^*P* < 0.05 vs. the DIR group.

**Figure 10:** Protein expression of Nrf2 and sulfiredoxin1 by western blotting (*n* = 4). The expression of Nrf2 and sulfiredoxin1 in lung grafts was measured by western blotting after 120 min of reperfusion in each group. (a) Representative bands of sulfiredoxin1, Nrf2, and *β*-actin; (b) expression of sulfiredoxin1 and Nrf2 normalized to *β*-actin. Nrf2: nuclear factor erythroid 2-related factor. In the DIRD group, the 3 *μ*g/kg of DEX was used. ^∗^*P* < 0.05 vs. the CS group; ^#^*P* < 0.05 vs. the DS group; ^△^*P* < 0.05 vs. the CIR group; ^§^*P* < 0.05 vs. the DIR group.

The article "Dexmedetomidine Alleviates Lung Oxidative Stress Injury Induced by Ischemia-Reperfusion in Diabetic Rats via the Nrf2-Sulfiredoxin1 Pathway" was published in 2022. Journal: Biomed Res Int.

**Figure 11:** Protein expression of Nrf2 and sulfiredoxin1 by western blotting in different concentrations of DEX groups (*n* = 4). The expression of Nrf2 and sulfiredoxin1 in lung grafts was measured by western blotting after 120 min of reperfusion. (a) Representative bands of sulfiredoxin1, Nrf2, and *β*-actin; (b) expression of sulfiredoxin1 and Nrf2 normalized to *β*-actin. Nrf2: nuclear factor erythroid 2-related factor. ^†^*P* < 0.05 vs. the DIR group; ^‡^*P* < 0.05 vs. the 3 *μ*g DIRD group; ^┼^*P* < 0.05 vs. the 5 *μ*g DIRD group.

**Table 1:** The indices of blood gas analysis (mean ± SD, *n* = 6).

	Group	T0	T1	T2	T3
PaO_2_/FiO_2_ (mmHg)	CS group	247 ± 2	245 ± 3	245 ± 2	247 ± 3
	DS group	245 ± 3	239 ± 2^∗^	234 ± 3^∗^	230 ± 1^∗^
	CIR group	245 ± 5	229 ± 3^∗^^#^	216 ± 2^∗^^#^	201 ± 2^∗^^#^
	DIR group	246 ± 1	224 ± 4^∗^^#△^	206 ± 5^∗^^#△^	184 ± 3^∗^^#△^
	DIRD group	247 ± 3	235 ± 4^∗^^#△§^	229 ± 4^∗^^#△§^	221 ± 3^∗^^#△§^

pH value	CS group	7.40 ± 0.01	7.40 ± 0.01	7.39 ± 0.01	7.40 ± 0.04
	DS group	7.39 ± 0.02	7.38 ± 0.01^∗^	7.37 ± 0.01^∗^	7.36 ± 0.02^∗^
	CIR group	7.40 ± 0.02	7.36 ± 0.01^∗^^#^	7.32 ± 0.01^∗^^#^	7.28 ± 0.01^∗^^#^
	DIR group	7.39 ± 0.02	7.34 ± 0.01^∗^^#△^	7.30 ± 0.03^∗^^#△^	7.24 ± 0.01^∗^^#△^
	DIRD group	7.40 ± 0.02	7.37 ± 0.01^∗^^#△§^	7.35 ± 0.01^∗^^#△§^	7.33 ± 0.01^∗^^#△§^

BE value (mmol/l)	CS group	0.07 ± 0.02	0.07 ± 0.03	0.09 ± 0.02	0.08 ± 0.03
	DS group	0.07 ± 0.03	−0.18 ± 0.04^∗^	−0.55 ± 0.12^∗^	−1.18 ± 0.15^∗^
	CIR group	0.06 ± 0.02	−1.05 ± 0.03^∗^^#^	−2.16 ± 0.22^∗^^#^	−2.57 ± 0.26^∗^^#^
	DIR group	0.07 ± 0.01	−1.61 ± 0.30^∗^^#△^	−2.81 ± 0.44^∗^^#△^	−3.85 ± 0.35^∗^^#△^
	DIRD group	0.08 ± 0.03	−0.60 ± 0.18^∗^^#△§^	−1.39 ± 0.34^∗^^#△§^	−1.86 ± 0.13^∗^^#△§^

PaCO_2_ (mmHg)	CS group	37.2 ± 4.0	40.2 ± 4.3	38.1 ± 4.1	40.0 ± 2.4
	DS group	49.6 ± 3.6	37.9 ± 2.5	39.0 ± 2.7	40.6 ± 2.6
	CIR group	36.8 ± 4.6	38.3 ± 4.0	40.8 ± 2.8	39.4 ± 3.1
	DIR group	36.7 ± 4.1	40.2 ± 4.9	36.7 ± 4.0	40.2 ± 3.8
	DIRD group	38.1 ± 2.5	37.8 ± 2.6	36.5 ± 4.3	39.2 ± 3.1

T0-T3 represented the baseline, 60 min after ischemia, and 60 min and 120 min after reperfusion, respectively. PaO_2_/FiO_2_: partial pressure of arterial oxygen (PaO_2_)/fraction of inspired oxygen (FiO_2_); BE: base excess; PaCO_2_: arterial carbon dioxide tension; CS: control+sham; DS: diabetes mellitus+sham; CIR: control+ischemia-reperfusion; DIR: diabetes mellitus+ischemia-reperfusion; DIRD: diabetes mellitus+ischemia-reperfusion+dexmedetomidine. In the DIRD group, the 3 *μ*g/kg of DEX was used. ^∗^*P* < 0.05 vs. the CS group; ^#^*P* < 0.05 vs. the DS group; ^△^*P* < 0.05 vs. the CIR group; ^§^*P* < 0.05 vs. the DIR group.

The article "Dexmedetomidine Alleviates Lung Oxidative Stress Injury Induced by Ischemia-Reperfusion in Diabetic Rats via the Nrf2-Sulfiredoxin1 Pathway" was published in 2022. Journal: Biomed Res Int.

**Table 2:** The indices of blood gas analysis from pulmonary vein (mean ± SD, *n* = 6).

	PvO_2_/FiO_2_ (mmHg)	pH value	BE value (mmol/l)	PvCO_2_ (mmHg)
CS group	248 ± 3	7.39 ± 0.02	0.10 ± 0.03	39.1 ± 1.6
DS group	228 ± 4^∗^	7.36 ± 0.02^∗^	−1.67 ± 0.23^∗^	39.3 ± 1.3
CIR group	198 ± 3^∗^^#^	7.28 ± 0.01^∗^^#^	−2.99 ± 0.31^∗^^#^	40.0 ± 1.2
DIR group	180 ± 3^∗^^#△^	7.24 ± 0.02^∗^^#△^	−4.21 ± 0.372^∗^^#△^	40.2 ± 1.4
DIRD group	218 ± 4^∗^^#△§^	7.33 ± 0.01^∗^^#△§^	−2.31 ± 0.25^∗^^#△§^	39.0 ± 1.4

PvO_2_/FiO_2_: pulmonary venous oxygen tension (PvO_2_)/fraction of inspired oxygen (FiO_2_); BE: base excess; CS: control+sham; DS: diabetes mellitus+sham; CIR: control+ischemia-reperfusion; DIR: diabetes mellitus+ischemia-reperfusion; DIRD: diabetes mellitus+ischemia-reperfusion+dexmedetomidine. In the DIRD group, the 3 *μ*g/kg of DEX was used. ^∗^*P* < 0.05 vs. the CS group; ^#^*P* < 0.05 vs. the DS group; ^△^*P* < 0.05 vs. the CIR group; ^§^*P* < 0.05 vs. the DIR group.

**Table 3:** Oxidative stress indices (mean ± SD, *n* = 6).

	8-OHdG (ng/ml supernatant)	MDA (nmol/mg protein)	iNOS (IU/ml supernatant)	GSH-PX (*μ*mol/mg protein)	SOD (U/mg protein)	T-AOC (U/mg protein)
CS group	0.69 ± 0.03	3.45 ± 0.23	187.3 ± 5.3	5.54 ± 0.28	94.9 ± 2.1	2.27 ± 0.13
DS group	0.74 ± 0.02^∗^	4.51 ± 0.33^∗^	202.1 ± 5.7^∗^	4.94 ± 0.13^∗^	85.2 ± 4.8^∗^	1.84 ± 0.07^∗^
CIR group	0.82 ± 0.04^∗^^#^	8.81 ± 0.60^∗^^#^	220.1 ± 3.9^∗^^#^	2.73 ± 0.15^∗^^#^	58.3 ± 2.2^∗^^#^	1.19 ± 0.06^∗^^#^
DIR group	0.88 ± 0.03^∗^^#△^	10.13 ± 0.46^∗^^#△^	234.0 ± 5.8^∗^^#△^	2.21 ± 0.13^∗^^#△^	40.7 ± 1.4^∗^^#△^	0.89 ± 0.03^∗^^#△^
DIRD group	0.77 ± 0.01^∗^^#△§^	5.22 ± 0.19^∗^^#△§^	210.7 ± 7.7^∗^^#△§^	3.25 ± 0.15^∗^^#△§^	78.5 ± 3.3^∗^^#△§^	1.55 ± 0.09^∗^^#△§^

8-OHdG: 8-hydroxydeoxyguanosine; MDA: malondialdehyde; iNOS: inducible nitric oxide synthase; GSH-PX: glutathione peroxidase; SOD: superoxide dismutase; T-AOC: total antioxidative capabilities; CS: control+sham; DS: diabetes mellitus+sham; CIR: control+ischemia-reperfusion; DIR: diabetes mellitus+ischemia-reperfusion; DIRD: diabetes mellitus+ischemia-reperfusion+dexmedetomidine. In the DIRD group, the 3 *μ*g/kg of DEX was used. ^∗^*P* < 0.05 vs. the CS group; ^#^*P* < 0.05 vs. the DS group; ^△^*P* < 0.05 vs. the CIR group; ^§^*P* < 0.05 vs. the DIR group.

## Data Availability

The datasets used during the current study are available from the corresponding author on reasonable request.
